# Falling and Drowning Detection Framework Using Smartphone Sensors

**DOI:** 10.1155/2022/6468870

**Published:** 2022-08-12

**Authors:** Abdullah Alqahtani, Shtwai Alsubai, Mohemmed Sha, Veselý Peter, Ahmad S. Almadhor, Sidra Abbas

**Affiliations:** ^1^College of Computer Engineering and Sciences, Prince Sattam Bin Abdulaziz University, AlKharj, Saudi Arabia; ^2^Information Systems Department, Faculty of Management, Comenius University, Bratislava, Odbojárov 10 82005, Bratislava 25, Slovakia; ^3^College of Computer and Information Sciences, Jouf University, Sakakah, Saudi Arabia; ^4^Department of Computer Science, Comsats University, Sahiwal, Pakistan

## Abstract

Advancements in health monitoring using smartphone sensor technologies have made it possible to quantify the functional performance and deviations in an individual's routine. Falling and drowning are significant unnatural causes of silent accidental deaths, which require an ambient approach to be detected. This paper presents the novel ambient assistive framework Falling and Drowning Detection (FaDD) for falling and drowning detection. FaDD perceives input from smartphone sensors, such as accelerometer, gyroscope, magnetometer, and GPS, that provide accurate readings of the movement of an individual's body. FaDD hierarchically recognizes the falling and drowning actions by applying the machine learning model. The approach activates embedding, in a smartphone application, to notify emergency alerts to various stakeholders (i.e., guardian, rescue, and close circle community) about drowning of an individual. FaDD detects falling, drowning, and routine actions with good accuracy of 98%. Furthermore, the FaDD framework enhances coordination to provide more efficient and reliable healthcare services to people.

## 1. Introduction

Smart health is an emerging paradigm that uses various smart devices, such as sensors, actuators, and smartphones, to support collaboration with other entities to provide various services such as health monitoring, activity recognition, fall detection, and activity assessment [1–6]. Activity recognition aims to extend the likelihood that an individual can live independently in a smart environment with machine learning techniques [7, 8]. Moreover, monitoring the changes in daily human life maximizes their productive time and reduces the cost of the healthcare system in later life [9].

Falls may result in dire health consequences such as severe injuries and disabilities in humans or even deaths. Researchers developed some fall detection systems to support independent and secure living. Research studies revealed that most people remain unable to retain their initial position by themselves after a fall [10, 11]. Reliable and accurate fall detection and prevention systems for citizens may play an essential role in taking better care of them [12]. Similarly, another serious threat to a human being is drowning. According to the World Health Organization (WHO), drowning is the third leading cause of unnatural deaths worldwide, of almost 7% of all injury-related deaths [13]. There are an estimated 3,20,000320,000 cases of annual drowning-related deaths worldwide.

To overcome the risks of death, an autonomous and unobtrusive framework requires recognizing an individual's actions and supporting rescue services in a context-aware environment. This paper focuses on the falling and drowning detection framework through smartphone sensors by utilizing ambient intelligence because of these issues and challenges. The smartphone technologies provide an unobtrusive solution with various accelerometers, gyroscopes, magnetometers, and location sensors. All individual actions can be tracked through these sensors while keeping the smartphone in the pocket [14]. Furthermore, ambient intelligence (machine learning) plays a vital role in transforming those actions into meaningful information.

To the best of our knowledge, only scarce studies exist on drowning detection using smartphone sensors and ambient technology. However, some studies such as [10, 11, 15–17] exist that focus only on fall detection frameworks. This paper provides a context-aware approach that identifies falling, drowning, and daily life activities and generates alerts to care providers. We collected the first dataset of individuals' actions through the accelerometer, gyroscope, magnetometer, and GPS sensors while performing falling and drowning activities. Furthermore, we combine the existing falling and daily life activities data with the collected drowning data to achieve robustness and diversity. The below points highlight our contributions:

- Propose a novel hierarchical approach for detecting falling, drowning, and routine life actions using machine learning classifiers.
- Provide the novel self-collected drowning and daily life activities dataset combined with the standard fall detection dataset.
- Effectively achieve the detection rate of drowning, fall, and routine life actions with consistent performance.

The remainder of this paper is organized as follows.  Section 2 provides the related work.  Section 3 presents the background, and Section 4 describes our proposed approach. The implementation of the work and evaluation of the approach to smart home data are presented in Section 5. Finally, Section 6 summarizes the results and discusses future work.

## 2. Related Work

This section presents the research studies relevant to fall and drowning detection. Fall and drowning detection approaches can be generally classified into ambient-based, vision-based, and wearable devices-based approaches [18, 19]. Ambient-based fall detection systems are built using various pressure, vibration, sensing, and audio signals. Fall detection studies used Mel-frequency Cepstral Coefficient (MFCC) to identify the fall and ADL events by processing audio or sensing signals [16].

Fall and ADL events usually portray discrete vibration patterns, which is this system's fundamental approach. Vibration signals are stockpiled by pressure sensors (resistive, piezoresistive) [15, 20] which are helpful in fall detection and prevention systems. Infrared sensors [21] are another suitable choice for fall detection and prevention systems that recent researchers prefer. Both pressure and audio signals are generally used to detect fall events. However, audio-based methods possess superior performance to pressure-based approaches.

Ambient-based systems place sensors in individual rooms or indoors only, which import blind spots or dead spaces in fall detection and prevention systems due to their limited range. Moreover, ambient systems are influenced by the external environment, such as the falling of some other object in a room kept under monitoring, impacting these systems' accuracy and producing plenty of false alarms.

Cameras are widely used in surveillance monitoring systems, which are now being used in fall detection and prevention systems under vision-based approaches. Various studies have used cameras (RGB or depth cameras) to detect head trajectories, body shape changes, or body posture to detect and prevent fall events. A system using one camera relying on the K-Nearest Neighbors algorithm was proposed to detect fall events based on silhouette change over time [22]. Although it is easier to set up, this approach's accuracy is insufficient due to limited area coverage. Researchers have also proposed fall detection systems with multiple cameras installed to enhance the precision of fall event detection and overcome the narrow area coverage problem as highlighted in former studies [10]. The precision of the fall event detection systems could be further optimized using depth cameras by calculating the distance between the floor and the critical joints of the body of a person [11, 23]. However, vision-based systems rely on complex image processing and computer vision techniques and demand proper storage and computing capacity. Moreover, the cameras are fixed in some places like rooms or buildings, so this approach's applicability is limited to indoors only.

Wearable device-based approaches are being studied extensively, which may be further grouped into threshold-based systems, machine learning-based systems, and hybrid systems. The threshold-based approach has been applied in many fall detection and prevention systems. With this approach's help, fall events are detected by comparing collected data with the personal preference settings (threshold). The threshold-based approach might be further designated into static and adaptive threshold-based methods. The fixed threshold value approaches were presented using Euler angle and sum vector magnitude features to detect fall events from ADLs relying on the receiver operating characteristics curve [24, 25]. Another fixed threshold value study predicted fall events by analyzing collected data from the 3-axial accelerometer and gyroscope sensors [26]. An object has received angular velocity, and acceleration signals were checked against preferred threshold values to predict pre-fall events. The threshold value chosen for an algorithm may impact the system's accuracy. The higher threshold value may become the reason for missing fall problems, and on the other hand, a lower threshold value may trigger false alarms.

The adaptive threshold value-based fall event detection and prevention methods are devised to overcome fixed threshold value-based methods' pitfalls. In a study, researchers devised an adaptive threshold approach to detect fall events relying on a multivariate control chart [27]. This adaptive threshold approach showed high detection accuracy with an individual's historical data, which can be considered a person-specific method. A similar study [28] presented a pre-impact fall prevention method built on an adaptive threshold model with an automatic threshold value adjustment ability using the person's motion history. In another research effort, [29], different groups of persons based on age, gender, height, and weight, were observed to improve the precision of personalized threshold value-based fall detection systems.

In the machine learning-based approach, K-Nearest Neighbor (KNN), Hidden Markov Model (HMM), Support Vector Machine (SVM), Random Forest (RF), and Naïve Bayes (NB) are frequently used algorithms in fall event detection and prevention systems. An HMM-based fall identification algorithm was presented based on a triaxial accelerometer in which acceleration signals had been examined by applying Gaussian distributions of hidden states in training the model [30]. Fall event detection has also been carried out using CNN's [31] training models with three feature sets selected from collected data from cameras and wave radars. Researchers have used the SVM machine learning technique to detect fall events by training their proposed classifier based on extracted features from gathered data to form a Kinect sensor [32]. In similar studies, SVM-based [33, 34] pre-impact fall event detection systems were introduced. In another study, neural networks were developed [35] to avoid fall events. These studies have illustrated that the accuracy of machine learning-based fall detection systems is greater than threshold-based systems due to trained classifiers on extracted features. Researchers have widely researched fall detection systems based on the accelerometer sensor.

A comparison study was carried out to observe the performance of accelerometer-based fall detection algorithms [36]. The comparison conducted with varying falling velocity, thresholds, and other similar parameters on real-world data revealed that the performance is below par compared to their performance measured in simulated environments. Another accuracy comparison study [37] revealed that machine learning-based approaches outperformed threshold-based approaches. Threshold-based and ML-based approaches to fall detection have their merits and demerits. Threshold-based algorithms need fewer computational resources and are easy to implement but lack accuracy. ML-based approaches enhance fall event detection accuracy but demand high computational resources and storage capacity. Nowadays, researchers are developing hybrid approaches combining threshold-based and machine learning-based methods to take the combined benefits of both these approaches and boost the accuracy of fall detection and prevention systems. A voting algorithm was proposed based on threshold methods to predict an optimized threshold value for fall detection [38] and fall prevention systems [39]. In recent days, hybrid methods have been proposed, combining multiple techniques, like threshold with SVM [40], or threshold with kernel density estimation [41] to decrease the frequency of false alarms.

The built-in sensors in smartphones like gyroscopes, accelerometers, and magnetometers are suitable for implementing falling and drowning detection systems. Authors in [42] tri-axial accelerometers and gyroscope sensors were applied in data collection. Then the data is transmitted over a mobile device where an individual's actions are recognized using a clustering algorithm. A study [43] presented android-based fall detection and prevention systems from various aspects such as sensors, system architecture, fall detection algorithms, and their response time to detect a fall event. Another study [44] pointed out that smartphone-based fall detection and prevention systems depend on the placement of sensors and their sensing mechanism. Still, there is a need for more accurate, efficient, and reliable fall detection systems to save older adults' precious lives.

To the best of our knowledge, existing studies only focused on fall detection using smartphones, on-body sensors [15, 16], vision-based approaches [10, 11], and wearable devices [17]. However, no study focuses on drowning detection using unobtrusive technologies such as smartphone sensors. This paper focuses on drowning and fall detection, as both are hierarchical in nature and pattern.

## 3. Background

### 3.1. Definitions

In this section, first, we explain the definitions that we will use in the remainder of the paper. The falling and drowning detection model learns from the input data stream provided by the smartphone sensors to recognize an individual's current state. The input data stream presents the continuous movement of the smartphone fused as a tuple containing sensor reading (*a*_*x*_, *a*_*y*_, *a*_*z*_, *m*_*x*_, *m*_*y*_, *m*_*z*_, *g*_*x*_, *g*_*y*_, *g*_*z*_, long, lat, label). Where (*a*_*x*_, *a*_*y*_, *a*_*z*_ ∈ accelerometer), (*m*_*x*_, *m*_*y*_, *m*_*z*_ ∈ magnetometer), (*g*_*x*_, *g*_*y*_, *g*_*z*_ ∈ gyroscope), (long, lat ∈ GPS) sensors and (label ∈ Drowning, Falling, routine). We refer label as a state that an individual is currently in, such as drowning, when an individual is drowning in water, falling when an individual is falling, and routine, when an individual is doing daily life activities. We hypothesized that these complex and life-saving activities could be detected using the machine learning model's hierarchical nature. Keeping in mind our hypothesis, we propose a novel decision-based hierarchical model to recognize an individual's current activity.

### 3.2. Problem Setup and Algorithm

Next, we formalize the problem according to the actual working recognition of activities. Given that a feature matrix consisting of activity instances *i*_*ji*_ of activity *A*_*i*_ given as input to a learning model returns a label *L*^*A*_*i*_^ of the recognized (*i*_*ji*_)th instances. Algorithm 1 is the procedure that demonstrates our proposed algorithm. Suppose *D* represents the dataset containing instance *I*=*i*_1_, *i*_2_,…, *I*_*n*_. Let TL represent the target class labels predicted by the classifier and NTL denote the total target classes. IC represents each instance's class, and TC represents the count of total predicted labels belonging to each class CL. Each instance in *I* is given as input to the classification model for predicting drowning, falling, and routine life actions. Let the performance measure Accuracy (A), Precision (p), Recall (R), F-Score (F), Roc Curve (RC), Confusion Matrix (CM), Validation Accuracy (VA), Loss (L), and Validation Loss (VL).

## 4. Fall and Drowning Framework

Before predicting that an individual is drowning, FaDD first predicts that an individual is falling and is then allowed to predict the drowning instances. In this way, our system becomes more powerful and robust.

This section discusses the steps that form our framework's building blocks: data collection, feature extraction, and machine learning model.  Figure 1 expresses the taxonomy of our proposed approach. First, we use smartphone sensors (accelerometer, gyroscope, magnetometer, and GPS) to collect each movement's data during fall and drowning positions and individuals' locations. Then we extract the features of fall and drowning movement for the ML model and location features to identify the individual's physical location. Further, we use the ML model to recognize whether the individual is drowning or not. The below subsection describes all these modules in detail, such as Data Collection, Feature Extraction, ML Model, and Intelligent Agent. Algorithm 1 is the procedure that demonstrates our proposed algorithm.

We developed an Android framework responsible for detecting falling and drowning actions. We made this framework runnable for almost every type of Android-based smartphones. The Android operating system allows applications to read data from a smartphone's sensors.

### 4.1. Sensed Data

Our framework FaDD controls the data collection process to be saved into a database and then recognized. For this process, FaDD uses four smartphone sensors: Accelerometer, Gyroscope, Magnetometer, and GPS. FaDD first takes permission to access these sensors. Then it senses the data at the frequency of 5 samples per second, so we have 300 samples per minute. This frequency is fine enough to capture all required actions. As we have to take care of battery life, recent studies have shown that the sensor invoking frequency is between 10 − 50 samples per second. We take five volunteers' services for sensing the data. One is a specialized trainer, two are medium-level swimmers, and the two are low-level swimmers. All volunteer belongs to an age group of 23 − 45. According to [45], physical activities at age 19 are comparable to levels at age 60. Hence, we felt this age group is enough to capture all posture readings. They were asked to mimic the postures of falling and drowning individuals. The participants were asked to keep the smartphone in their pants pocket, as shown in the figure. To ensure the sensed data's quality, our co-author controls and monitors this task.

### 4.2. Cloud Database

After sensing the data through smartphone sensors, we use Google's cloud-based database Firebase to save the sensed data readings. The Firebase database gives more secure authentication, real-time response, and efficient performance. Since, privacy and security are one of the leading challenges of healthcare data [46, 47]. Furthermore, Firebase helps us send the data timely for pre-processing, feature extraction, and ML algorithms. Firebase can run in offline mode. Firebase re-sends any writes when network connectivity is restored.

### 4.3. Feature Extraction

The sensed data stored in the cloud database contains 12 features. This includes one time feature [Time], three-axis of accelerometer [*Ax*_1_, *Ay*_2_, *Az*_3_], three-axis of gyroscope [*Gx*_1_, *Gy*_2_, *Gz*_3_], three-axis of magnetometer [*Mx*_1_, *My*_2_, *Mz*_3_], and two-axis of GPS sensor [*l*at, long]. We extract the nine features of the three-axis accelerometer, gyroscope, and magnetometer as input to the ML model to predict the activity being performed. The output of the ML model is a label of activity. The time feature is converted into standard time to be sent at the notify step of FaDD. The two-axis features of GPS are converted into the participant's physical address to be sent in the future to notify emergency alert.

### 4.4. Machine Learning Model and Parameter Tuning

We apply three machine learning models: Logistic Model Trees (LMT), Bayes Net (BN), and Logistic Regression (LR) for drowning detection. We select these models based on their importance in covering the problem from all possible aspects. LMT combines decision tree and logistics regression to overcome a machine learning model's over-fitting problem. BN is a probabilistic model that uses the Bayesian method for probability computations, while LR uses a regression function to classify the test data. LR works best when the input variables are not correlated. These models are tuned according to the required results. Tuning maximizes a supervised machine learning model's classification performance without overfitting or producing too high a variance. According to our problem, LMT is used with a batch size of 50, and the beta for trimming the weight of Logitboost is set to 0. For Bayes-Net, we set the batch size to 100 and fast regression to True to get better results. LR is used for building and using a multinomial logistic regression model with a ridge estimator. We use the default parameters for LR.

### 4.5. Alert Notify

This framework step is a future idea to send an emergency alert about individuals' actions. Therefore, an alert mechanism could be embedded in the smartphone application after recognizing instances of sensed data such as falling and drowning. The alert mechanism will send an emergency alert to the android interface of the guardian, close circle community, and rescue bodies with the individual's location. In this way, an individual can get emergency aid, eventually reducing the unnatural death rate.

## 5. Experimental Results and Evaluation

This section discusses evaluating our proposed approach by analyzing the dataset. We collect the labeled data to train the Machine Learning (ML) model. Three ML models Logistic Model Trees (LMT), Bayes Net (BN), and Logistic Regression (LR), are used to recognize the drowning, routine, and fall activities. We also make a customized setting with parameter tuning of these models. We apply five-fold cross-validation for all experiments. It works by leaving the 1 : 5 part of the data for testing and using the 4 : 5 part of the data for training.

### 5.1. Dataset

We collected a large and diverse labeled dataset to train and test the ML model. Data is collected from five participants for falling and drowning activities. The participants were asked to keep the smartphone in their pants pocket.  Figure 2 demonstrates the different diverse postures we follow to collect the data on drowning and falling actions. Through four smartphone sensors: accelerometer, gyroscope, magnetometer, and GPS, the dataset contains 12 features. The nine features of 3 axis accelerometer, gyroscope, magnetometer, two features of GPS, and one label feature are used for training and testing the ML model. The usage of the other three features is discussed in Section 4.3. It collects the data at the frequency of 5 samples per second, so we have 300 samples per minute. The data collection duration was approximately 13–18 minutes for each participant. This task was controlled and monitored by our co-author to ensure the quality of the data. As our approach is hierarchical. We collected the data on falling and drowning.

We also use the data of the other 15 types of daily life activities stated in the study [48]. Although their dataset contains many examples of all 15 types of activities, we only use almost 1000 random examples of each activity. We label these examples routine activities to avoid intra-class problems between these 15 activities. The rationale behind collecting this data is that as drowning is a serious problem, and the framework should not directly classify instances as drowning and alert the nearby help center. Therefore, we use the data of these daily life activities to make a clear and robust recognition of drowning, falling, and regular activities. We got 11091 samples of drowning activity in data collection, 11700 samples of routine activity, and 6548 samples of falling activity.  Table 1 demonstrates the details of the dataset.

Table 2 present the details of the statistics of activity occurrence frequencies.

### 5.2. Data Analysis

This section analyzes the variations of each axis of the accelerometer, gyroscope, and magnetometer sensor. These variations depict human physical movements. Due to less gravity underwater, the gyroscope does not provide helpful information. Therefore, we removed thissensordata from thefinal dataset. Figures 3–5 depicts the data samples of an accelerometer, a gyroscope, and magnetometer sensors and their corresponding spectrum. These samples belong to 3 activities: falling, drowning, and routine daily life activities, where the variation of drowning activity lies in the range of [−20,41], and the variation of falling activity lies in the range of [−38,50], and the variation of routine activity lies in the range of [−60,110].

Figure 3 reveals interesting essential information about the directions of falling activity. For falling activity, the accelerometer and magnetometer signal are not subtle. Blue Spikes correspond to the acceleration in a positive direction continuous in the entire vector, and similar is for the *Ay*-axis. The *Z*-axis of the accelerometer is the major contributor to detecting a fall as there is a sudden spike at the 71th − 76th instances depicting a person's fall. The magnetometer is crucial for detecting the device's orientation relative to the Earth's magnetic north. Here *Mz* shows the direction of activity from point *X* to point Y. When a person fell, the magnetometer's *MxAxis* produced a sudden spike in the positive direction, and *My* produced a spike in the negative direction towards the Earth. It is worth noticing that the gyroscope is not helpful for fall detection as it produces continuous flat signals.

For drowning activity, the accelerometer and magnetometer signal is usually subtle.  Figure 4 reveals interesting essential information about the directions of drowning activity. All three axes of the accelerometer and magnetometer are continued and do not show periodic spikes in the selected vector. For drowning activity, the accelerometer and magnetometer signal is subtle. When a person falls in the water, the position of the leg sometimes moves upward and downwards. The *My* axis of the magnetometer produced a sudden spike in the positive direction, and *My* produced a spike in the negative direction towards the Earth, which can help predict the drowning of a person.

For falling activity, the accelerometer and magnetometer signal are not subtle as it provides periodic behavior of spikes going upwards and downwards for all the sensors as shown in Figure 5. These signals were captured while a participant performed daily life tasks such as walking, eating, toileting, etc. It is worth noticing that a machine learning model can learn the boundaries of each three activities considered in this paper as they are pretty distinctive.

### 5.3. Evaluation Metrics

Evaluation metrics are a necessity to assess the performance of the ML model. Almost all evaluation metrics depend on the nature of the dataset. Usually, the accuracy is taken as a primary metric to check the ML model's performance, but the dataset is balanced. However, when the dataset contains unequal classes, it does not provide valuable information. Thus, We extract results by accuracy, recall, precision, and f-score metrics to ensure the model's reliability. We extract results on different evaluation metrics for further comparison. Below, we show the equations and definitions of evaluation metrics. Further, we also extract the confusion matrix to show how many examples of one activity are wrongly recognized as an example of other activities.

Accuracy shows the overall recognition rate of the ML model. It is calculated using True Positive (TP): correctly recognized samples, True Negative (TN): examples of other activities correctly recognized as one activity example, False Positive (FP): examples of other activities wrongly recognized as one activity examples, and False Negative (FN): examples wrongly recognized as other activities examples as shown in (1)

(1) $$\begin{array}{c} \text{Accuracy}=\frac{\text{TP}+\text{TN}}{\text{TP}+\text{TN}+\text{FP}+\text{FN}}. \end{array}$$

Recall shows the correctly predicted examples of one activity from all the examples. The recall is also known as the sensitivity of the ML model. It is calculated using TP and FN as shown in (2)

(2) $$\begin{array}{c} \text{Recall}=\frac{\text{TP}}{\text{TP}+\text{FN}}. \end{array}$$

Precision shows the correctly predicted examples of one activity from all the predicted examples. Precision is also called positive predictive value. It is calculated using TP and FP as shown in (3)

(3) $$\begin{array}{c} \text{Precision}=\frac{\text{TP}}{\text{TP}+\text{FP}}. \end{array}$$

F-score is computed as the harmonic mean of recall and precision as shown in (4)

(4) $$\begin{array}{c} F-\text{Score}=2\times \frac{\text{Precision}\times \text{Recall}}{\text{Precision}+\text{Recall}}. \end{array}$$

## 6. Results

Figure 6 demonstrates the precision metric on drowning, regular, and falling activities using LMT, BN, and LR ML models. It shows that the LMT and BN achieve 25% better precision than LR on drowning activity. In the case of routine activity, LMT achieves 3% and 38% better precision than BN and LR. While, on falling activity, LMT achieves 11% and 30% better precision than BN and LR. The BN achieves 25%, 33%, and 19% better precision than LR on drowning, regular, and fall activities, respectively.

Figure 7 demonstrates the recall metric for drowning, routine, and falling activities using LMT, BN, and LR ML models. It shows that the LMT achieves 4% and 23% better recall than BN and LR on drowning activity. In the case of routine activity, LMT achieves 4% and 34% better recall than BN and LR. While, on falling activity, LMT achieves 4% and 36% better recall than BN and LR. The BN achieves 19%, 30%, and 32% better recall than LR on drowning, regular, and fall activities.

Figure 8 demonstrates the f-score metric on drowning, routine, and falling activities using LMT, BN, and LR ML models. It shows that the LMT achieves 3% and 25% better f-score than BN and LR on drowning activity. In the case of regular activity, LMT achieves 2% and 33% better f-score than BN and LR. While, on falling activity, LMT achieves 9% and 35% better f-score than BN and LR. The BN achieves 22%, 31%, and 26% better f-score than LR on drowning, regular, and fall activities.

Figure 9 demonstrates the accuracy metric on drowning, routine, and falling activities using LMT, BN, and LR ML models. It shows that the LMT achieves 4% and 23 better accuracies than BN and LR on drowning activity. In the case of regular activity, LMT achieves 4% and 34% better accuracy than BN and LR. While, on falling activity, LMT achieves 4% and 36% better accuracy than BN and LR. The BN achieves 19%, 30%, and 32% better accuracy than LR on drowning, regular, and fall activities.

Figure 10 presents the confusion matrix on drowning, routine, and falling activities using the LMT model. It shows that less than 1% example of drowning activity is wrongly recognized as examples of routine and fall activities. In the case of regular activity, only 1% examples were wrongly recognized as examples of fall activities. Simultaneously, only 2% examples of falling activity are wrongly recognized as examples of routine activities.

Figure 11 presents the confusion matrix on drowning, routine, and falling activities using the BN model. It shows that only 1% and 3% examples of drowning activity are wrongly recognized as examples of routine and fall activities. Also, only 1% and 5% examples of regular activity are wrongly recognized as examples of drowning and fall activities. At the same time, 1% and 5% examples of falling activity are wrongly recognized as examples of drowning and routine activities.  Figure 12 presents the confusion matrix on drowning, routine, and falling activities using the LR model. It shows that only 35% and 1% examples of drowning activity are wrongly recognized as examples of routine and fall activities. In the regular activity, 20% and 16% examples are wrongly recognized as examples of drowning and fall activities. Simultaneously, 12% and 26% examples of falling activity are wrongly recognized as examples of drowning and routine activities.

## 7. Conclusion and Future Work

Falling and drowning are underlined reasons with an almost 7% death rate of overall unnatural deaths. Detecting falling and drowning is more challenging than other activities since cameras and sensors cannot be installed everywhere. To overcome these challenges, this paper presented a novel, unobtrusive, ambient intelligent framework, Falling and Drowning Detection (FaDD). FaDD is the first, unobtrusive framework that uses smartphone sensors to depict an individual's body's readings and recognize them using ML algorithms as falling, drowning, and routine actions. FaDD achieves a 98% of accuracy. The limitation of this study is that WiFi and other cellular signal does not work properly underwater. FaDD presents the emergency alert mechanism as an abstract idea that could address in the future. The emergency alert mechanism generates an emergency alert with an individual's location to its guardian, close circle community, and rescue team to save an individual. The FaDD framework will enhance coordination to provide more efficient and reliable healthcare services to people. In the future, researchers can use smart watches and other on-body sensors to overcome these limitations.

## Figures and Tables

**Figure 1:** Taxonomy of proposed approach for falling and drowning detection.

**Figure 2:** Data collection postures of the falling and drowning activity.

**Figure 3:** Sensor variations of falling activity.

**Figure 4:** Sensor variations of drowning activity.

**Figure 5:** Sensor variations of routine activity.

**Figure 6:** Comparison of Precision of LMT, BN, and LR classifiers.

**Figure 7:** Comparison of recall of LMT, BN, and LR classifiers.

**Figure 8:** Comparison of F-score of LMT, BN, and LR classifiers.

**Figure 9:** Comparison of accuracy of LMT, BN, and LR classifiers.

**Figure 10:** Confusion matrix using the LMT model.

**Figure 11:** Confusion matrix using the BN model.

**Figure 12:** Confusion matrix using the LR model.

**Algorithm 1:** Algorithm for the Falling and Drowning Framework.

**Table 1:** Characteristics of the dataset and devices.

Parameter	Value
Smartphone	Samsung galaxy S10
Smart phone type	Waterproof
Sensors readings	Accelerometer, gyroscope, magnetometer, GPS
Dataset name	Falling and drowning
Dataset type	Self collected
Number of participants	5
Mean age	26
Total main activities	3
Activity 1	Drowning
Activity 2	15 daily life activities (routine)
Activity 3	Falling

**Table 2:** Summary statistics of activity occurrence frequencies for the developed dataset used in our paper.

Feature	Minimum	Maximum	Mean	Standard deviation
*Ax*	−32.741	32.737	−1.532	6.787
*Ay*	−32.732	32.756	−1.084	6.728
*Az*	−32.765	32.767	−1.15	7.47
*Gx*	−22.521	21.634	−0.057	1.208
*Gy*	−29.202	29.548	−0.078	2.407
*Gz*	−28.638	27.36	0.075	1.903
*Mx*	−55.875	52.875	5.088	27.911
*My*	−55.438	53.75	15.224	22.385
*Mz*	−52.75	53.75	16.44	25.485

## Data Availability

The Fall and Detection dataset used to support the findings of this study is available from the corresponding author upon request.
